The article "Single and Combined Neuroimaging Techniques for Alzheimer's Disease Detection" was published in 2021. Journal: Comput Intell Neurosci.

# Single and Combined Neuroimaging Techniques for Alzheimer's Disease Detection

**DOI:** 10.1155/2021/9523039

**Published:** 2021-07-13

**Authors:** Morteza Amini, Mir Mohsen Pedram, Alireza Moradi, Mahdieh Jamshidi, Mahshad Ouchani

**Affiliations:** ^1^Department of Cognitive Modeling, Institute for Cognitive Science Studies, Shahid Beheshti University, Tehran, Iran; ^2^Department of Electrical and Computer Engineering, Faculty of Engineering, Kharazmi University, Tehran, Iran; ^3^Department of Cognitive Modeling, Institute for Cognitive Science Studies, Tehran, Iran; ^4^Department of Clinical Psychology, Faculty of Psychology and Educational Science, Kharazmi University, Tehran, Iran; ^5^Department of Cognitive Psychology, Institute for Cognitive Science Studies, Tehran, Iran; ^6^Department of Mathematical Sciences, Faculty of Mathematical Sciences, Shahid Beheshti University, Tehran, Iran; ^7^Institute for Cognitive and Brain Science, Shahid Beheshti University, Tehran, Iran

## Abstract

Alzheimer's disease (AD) consists of the gradual process of decreasing volume and quality of neuron connection in the brain, which consists of gradual synaptic integrity and loss of cognitive functions. In recent years, there has been significant attention in AD classification and early detection with machine learning algorithms. There are different neuroimaging techniques for capturing data and using it for the classification task. Input data as images will help machine learning models to detect different biomarkers for AD classification. This marker has a more critical role for AD detection than other diseases because beta-amyloid can extract complex structures with some metal ions. Most researchers have focused on using 3D and 4D convolutional neural networks for AD classification due to reasonable amounts of data. Also, combination neuroimaging techniques like functional magnetic resonance imaging and positron emission tomography for AD detection have recently gathered much attention. However, gathering a combination of data can be expensive, complex, and tedious. For time consumption reasons, most patients prefer to throw one of the neuroimaging techniques. So, in this review article, we have surveyed different research studies with various neuroimaging techniques and ML methods to see the effect of using combined data as input. The result has shown that the use of the combination method would increase the accuracy of AD detection. Also, according to the sensitivity metrics from different machine learning methods, MRI and fMRI showed promising results.

## 1. Introduction

Alzheimer's disease (AD) can be considered a gradually progressive neurodegenerative disease process that involves gradual synaptic integrity and loss of cognitive functions [1]. Early detection of AD will help to prevent catastrophic damage to the brain. One of the most significant signs and biomarkers for AD are beta-amyloid, tau protein, and miRNA [2]. This marker has a more critical role for AD detection than other diseases because beta-amyloid can extract complex structure form [3]. Detecting biomarkers deposition and brain structure examination with neuroimaging techniques like functional magnetic resonance imaging (fMRI) and positron emission tomography (PET) approaches have been widely exploited nowadays. Amyloid PET was used to determine brain amyloid plaque load scores as a biomarker [4]. Observation of fMRI techniques will help detect dementia and change in neuron connections, determining the change in brain function. On the other hand, the level of amyloid deposition in certain parts of the brain, which can be seen by amyloid PET biomarker, will help to survey AD severity for patients [5]. However, especially in cases of dementia diagnosis, mentioned biomarkers could not help accurately identify or predict cognitive deterioration due to individual threshold differences in each subject [6]. The use of PET for AD detection will consume more time, and because of isotope injection, it is considered an invasive technique. MRI and its branches like fMRI for AD detection and classification are other areas of research in neuroimaging. For the change in structure detection use of the fMRI technique is more convenient than other neuroimaging techniques.

The article "Single and Combined Neuroimaging Techniques for Alzheimer's Disease Detection" was published in 2021. Journal: Comput Intell Neurosci.

The better change in brain detection structure using structural magnetic resonance imaging (sMRI) can help. Suppose that, with the survey of sMRI, enough structural features have not been extracted. In that case, resting-state fMRI (rs-fMRI) can provide more valuable and complementary information to distinguish early-stage dementia and AD detection in each patient [7]. Combining fMRI and PET into one unique scanner has allowed the researcher to explore the underlying neurochemistry of brain function in more detail [8]. A combination of PET and fMRI techniques resulted in spatial and quantifiable inconsistencies as active data acquisition. By the combination of PET and fMRI, Wehrl et al. [9] extracted functional connectivity of the subjected rat brain. In a nutshell, the fMRI technique will help extract nine well-known biological neural networks in brain structure.

In contrast, the PET technique identified seven glucose metabolism-related biological networks. Different studies have shown comprehensive and complementary information using combination techniques to decode brain function and brain networks further, so that the question of which brain neuroimaging technique will be more helpful and practical for Alzheimer-related disease (ARD) detection and classification arises. In this research, we focus on different branches of AI (artificial intelligence) like machine learning (ML) and deep learning (DL) algorithms for ARD prediction with PET, fMRI, sMRI, and combination methods. Increasing the number of patients with AD-related problems in the future is inevitable. It has been estimated that 1 of 85 individuals in 2050 would suffer from AD-related disease, so, with growth in the number of patients with AD-related problems [10] and with new corona virus pandemics emergence in 2019, different studies have categorized patients with neurodegeneration problems like AD, mild cognitive impairment (MCI), and other ARD at high risk for COVID-19 [11]. Different stages of AD and its complications will be associated with high morbidity and mortality rate. ARD will cause memory capacity loss. Most Alzheimer's patients will forget how to correctly conduct the recommendations from public health authorities or World Health Organization (WHO) to reduce the COVID-19 spread in a high-risk community.

The article "Single and Combined Neuroimaging Techniques for Alzheimer's Disease Detection" was published in 2021. Journal: Comput Intell Neurosci.

For example, WHO's known recommendations are constant hand washing, covering mouth and nose when coughing or sneezing, monitoring physical and temperature conditions for reporting symptoms of COVID-19, and preserving at least 6 ft physical distance from other people, especially elderly peoples [11]. This specific order is crucial to AD patients, especially when considering these people's age groups, which usually are more than 65 years. Even patients with MCI or milder dementia may forget to conduct these procedures due to oblivion or depression. Those with more severe dementia cannot correctly comprehend or remember most of these orders due to the strictness of their short-term memory.

Another complication of ARD consists of financial problems. Single Medicare beneficiaries diagnosed with ARD have a higher probability of missing payments on credit accounts. These negative financial consequences continued after the progress of ARD and will cause 10% to 15% of missed payments. These financial complications from AD were common in none of the educational college groups [12]. With this significant complication, proper and fast detection of Alzheimer in the early stages will help patients prevent financial and physical complications. ML and DL algorithms for ARD classification and detection have gained much attention in the past decade. With the growth in computational power and emergence of more sophisticated and supervised algorithms like convolutional neural network (CNN) development of artificial intelligence (AI) application in healthcare has increased rapidly [13, 14]. All artificial intelligence models will use some training data such as pictures from neuroimaging techniques and other electronic healthcare data to extract full features or direct samples to classify, detect, and recognize ARD. Numerous ML applications involve tasks that can be set up as supervised and semisupervised learning [15]. ML algorithms often have reached more than 96% to classify AD [16, 17]. This state-of-the-art result for binary classification of AD is no surprise due to the structure of DL algorithms and the usage of neuroimaging data. Proper preprocessing of input data into the balance group of data mentioned result is no longer a surprise. Nevertheless, the vacancy of specific research on the effect of single and combined neuroimaging techniques for reaching the mentioned results and comparing them is increasing. This paper reviewed AD detection, early recognition, and classification using different machine learning applications with fMRI, PET, sMRI, and combined neuroimaging techniques.

The article "Single and Combined Neuroimaging Techniques for Alzheimer's Disease Detection" was published in 2021. Journal: Comput Intell Neurosci.

## 2. Data Set

Brain imaging gathering procedure can be categorized as noninvasive like fMRI and sMRI techniques or invasive techniques like PET. For example, rs-fMRI is a neuroimaging technique commonly used to study the progressive and pathogenic procedure of neurodegeneration diseases like AD. Other techniques we have surveyed in this article impacted the brain's specific marker or specific area. All images presented in this paper were obtained from the Alzheimer's Disease Neuroimaging Initiative (ADNI) repository, which can be found at https://www.loni.ucla.edu/ADNI and https://www.adni-info.org. The ADNI database contains 1.5 T and 3.0 T t1w MRI scans for AD, MCI, and cognitively normal conditions in various patients with different ethnic groups. This repository offers data as the image for three categories of patients: NC, AD, and MCI. These three categories will comprise the whole condition of each patient in this research.

### 2.1. MRI

This data gathering technique will use radio waves and magnetic fields to acquire compelling images with high discriminative features and high-resolution images. This technique can return 2D and 3D images of brain structures with high quality. This technique would not use any harmful radiations from X-rays or other radioactive tracers, so it will be categorized as a noninvasive and nonharmful neuroimaging technique. The most used MRI techniques for AD detection and classification comprise sMRI, which helps technicians evaluate brain volumes in pictures to detect brain loss of tissue, cells, neurons, and other destructive changes. Brain degeneration is an unavoidable component of ARD that causes memory loss and self-unawareness in patients [18].  Figure 1 shows an example of an MRI picture which has been used to detect brain decrease in tissue. In a nutshell, the MRI technique will exploit the nucleus of hydrogen atoms as small magnets as a tracer [19]. Then the vibration of this nucleus of hydrogen atoms can be manipulated to become a tracer and generate a signal that will turn into an image.

The article "Single and Combined Neuroimaging Techniques for Alzheimer's Disease Detection" was published in 2021. Journal: Comput Intell Neurosci.

### 2.2. fMRI

fMRI can be categorized as noninvasive technique because this technique focuses on measuring and mapping brain activities without any injected tracer to patients' bodies. With the change in the body's activity, neuron activity in the brain constantly fluctuates [20]. This technique is also using the effect of magnetic fields on brains in order to gather data. The cylindrical tube of an MRI scanner houses a potent electromagnet field, which will be used to gather information whereas patients are conducting some activities. As it has been told before, this strong field will affect the magnetic behavior of atoms. Typically the atomic nuclei orientation is stochastic and does not create any specific pattern. However, under the encouragement of a magnetic field, the pattern of nuclei becomes allied with the direction of the field and makes a specific pattern. As stronger magnetic field becomes significant, the effect will be on the nuclei and degree of alignment. At last, with these powerful aligned signals from these individual nuclei, measurements of these pales will be possible. In fMRI neuroimaging techniques, the behavior of magnetic signal from the core of hydrogen atoms in a water molecule is detected as a tracer. The different neural activity of the body of different parts of the brain will increase; therefore, an improvement in demand for oxygen will be generated (see Figure 2).

With high blood pressure and movement of the capillary blood cells, the local response in a different part of the brain will increase biological neural activity. Red blood cells have hemoglobin. Hemoglobin is diamagnetic when it conveys oxygen in blood and paramagnetic when it conveys carbon dioxide [21], for gathering MRI picture. This difference in magnetic properties will be practical to use. As it has been said before, since the amounts of oxygen that each blood cell will transform will be different according to the different levels of biological neural activity in the brain, these can be used as markers to detect brain activity. A sample of fMRI pictures containing 64 different images of a patient was surveyed in this research. The fMRI picture of the brain is shown in Figure 2. So, with gathering different parts of the brain, brain structure will be revealed, and with different actions in the body like the movement of arms or feet, different parts of the brain will be activated and can be seen in the fMRI scans.

The article "Single and Combined Neuroimaging Techniques for Alzheimer's Disease Detection" was published in 2021. Journal: Comput Intell Neurosci.

The use of fMRI scans for AD detection was widely used last decade [22, 23]. A different part of brain activity can be discriminated even from a different view with this image. Some pictures from a different region of the brain are shown in Figure 3.

### 2.3. rs-fMRI

rs-fMRI focuses on low-frequency that is defined as less than 0.1HZ impulsive fluctuations in the level of blood cells that carry oxygen in the brain section. The whole procedure of data gathering rs-fMRI occurs when a patient is at rest situation [24]. The main key characteristic in rs-fMRI was synchronism of low-frequency fluctuations in the tracer signal arising from the right and left primary motor regions of cortices at rest condition of each patient for surveying. With this neuroimaging technique, most researchers have reached a connectivity pattern that is sufficiently close to the activation pattern from a two-sided finger-tapping task [25]. It extracted abnormal patterns in the resting situation of each patient. It disrupted connectivity in various parts of biological neural networks so the brain can help clarify some of the motor and nonmotor shortfalls seen in patients with ARD [26]. A sample of the rs-MRI picture is shown in Figure 4. This picture contains 54 stages of patients in resting condition. The size of samples in this figure is 256*∗*64.

So, with different stages of the brain, even in resting conditions, different patterns can be exploited to classify AD patients.

### 2.4. PET

PET is the most exact and delicate neuroimaging technique for capturing the molecular image, which helps extract communications and pathways within humans' brains [27]. The specificity rises from the variety of positron-emitting radionuclides choice, which can be defined as specific biomarkers for pathway recognition, biochemicals, and pharmaceuticals without disturbing their biological function [28]. Furthermore, the radiation used as a radiolabeled tracer can be sensed when the reflect wave has been reported above the low natural radiation background. The initial provocation for PET use was for human brain studies. Researchers have used PET for gathering anatomical and biological complexity from brain organs. Because of the use of injected tracer in this procedure, this technique will be considered an invasive method [29]. The compassion and chronological resolution of PET scanners provided to researcher scans with kinetical features that constants of neurotransmitter pathways and binding could be extracted from correct input data [30]. The main concern of the PET technique is to gather more high-quality pictures with better discriminative spatial resolution features and increased axial coverage. With the success of this technique, most researchers worldwide have used this picture for regional brain activation detection. PET pictures are sometimes helping to detect diseases like Alzheimer's faster than other imaging procedures [31]. Some samples of PET with 336*∗*336 are shown in Figure 5. As it has been shown in Figure 5, these PET pictures have more different stages than fMRI or rs-fMRI.

The article "Single and Combined Neuroimaging Techniques for Alzheimer's Disease Detection" was published in 2021. Journal: Comput Intell Neurosci.

Here the number of different pictures has reached 654. This increase in pictures will cause better observation and PET's image will become more conventional. However, as said before, capturing all of these pictures can lead to 4 to 6 hours of tedious procedure. Also, this neuroimaging technique is invasive [32]. The most used case of PET is to survey the chemical activity in the brain tissue of each subject. These neuroimaging techniques will help to determine the different conditions of each patient, which include brain disorders. The pictures from a PET scan provide diverse data which are uncovered by other kinds of neuroimaging techniques, like computerized tomography (CT) or MRI. A PET scan or a combined CT-PET scan enables neuroscientists to identify illness and measure the condition of the brain of each patient more conveniently. PET images nowadays will be recorded by about 1% of the equivalent couples of photons emitted from the brain of each subject and the learned coincidences data from each patient. This data will be stored in list mode as separate events with a time brand or sorted into arrays, sinogram. Then, using this data cluster of tracers 3D distribution of the tracer can be recreated [33] (see Figure 6).

## 3. Combination of PET and MRI Techniques

MRI and PET techniques have opposite natures for gathering data from the brain. By combining these neuroimaging techniques, more accurate AD diagnosis or classification tasks can be conducted [34]. In Figure 6, a combination of PET and rs-fMRI has been shown. New researches show that a mixture of one or more biomarkers may deliver complementary material for ARD diagnosis; also, combination data can help to increase the classification accuracy. This combination of biomarkers can be presented as fluorodeoxyglucose positron emission tomography (FDG-PET), sMRI, cerebrospinal fluid (CSF) protein levels, and apolipoprotein-E (APOE) genotype [35]. Although published approaches based on the combination of techniques have applied dissimilar biomarkers to develop a new neuroimaging biomarker for AD, this usage of combination methods may be limited [36]. The usage of combination techniques has led to early detection in some approaches [36]. Based on the performance of ensemble learning models and multikernel learning success on combination neuroimaging techniques in the last decade, these techniques are popular for AD detection and classification [37, 38]. The combining method showed promising results and can be considered the future of AD detection and classification input data, especially in early detection cases [39, 40].

The article "Single and Combined Neuroimaging Techniques for Alzheimer's Disease Detection" was published in 2021. Journal: Comput Intell Neurosci.

### 3.1. Combination Method Preprocessing

After gathering different data set use of various preprocessing procedures is necessary for better prediction of results. As it has been said before use of a combination of neuroimaging techniques has resulted in better classification and detection of ARD. Methods like Dartel are considered preprocessing procedures for combination input data. Dartel is a proper tool for increasing intersubject recording or three-dimensional normalization of functional and structural scans, providing less flattening and improving MRI-PET combination data [41]. Another approach has worked on a framework based on an early union procedure that uses different combination rules to combine opposite data from different biomarker modalities into a single feature vector [42]. In another research, they focused on region of interest (ROI) for gathering complementary information of each neuroimaging method. Many researchers used data from the ADNI database and divided brains based on two atlases: LONI Probabilistic Brain Atlas and Automated Anatomical Labeling. Then baseline images of sMRI and 18F-fluorodeoxyglucose PET were used to calculate average gray-matter density and average relative cerebral metabolic rate for glucose in each region [43]. In 2008 compatible PET detector tools for gathering synchronized PET/MR images of the human brain were conducted. With these new tools and new studies, researchers successfully achieved brain glucose consumption images in two subjected patients using 18F-FDG-PET, MR imaging, and MR spectroscopy [44]. With the combination of data, they established that PET/MR imaging combination is possible in humans' brains. With this combination of data for the first time, a field of new possibilities in molecular imaging areas and ARD detection have been unlocked. The essential step of combination techniques and preprocessing methods is shown in Figure 7. A typical pipeline for the combination of PET with rs-fMRI is shown in Figure 7.

In the first step, frontal commissure and subsequent commissure correction for all subject images can be extracted with this combination of data. After data gathering use of N4 bias field correction using ANT's toolbox will help correct the intensity of nonhomogeneity for each patient's image [45]. In some cases, elimination of skull has been conducted, which was unnecessary if images were already preprocessed. For the MRI images, aligning them to the MNI152 T1-weighted standard image using a standard procedure will be done next. In normalization steps, the extracted features will throw a standard scalar function, which transforms the array of input matrix data sets into a standard distribution with minimum and maximum of each column vector, which can help to reduce the redundancy and dependency of the data [46]. For structural and functional segmentation of brain into the anatomical area and enumerating these extracted features from each specific ROI from each sMRI image, toolbox with a conventional procedure like NiftyReg with 2 mm Brainnetome Atlas template has been used [47]. After gathering ROI from labeled sMRI images, computed volume of gray-matter tissues in that ROI will be used as an input feature for the detection task.

The article "Single and Combined Neuroimaging Techniques for Alzheimer's Disease Detection" was published in 2021. Journal: Comput Intell Neurosci.

### 3.2. Single Method Preprocessing

For processing fMRI pictures into using robust data for early MCI detecting, a handful of researchers have used Data Processing Assistant for Resting-State (or in brief DPARSF) [48–51]. To process fMRI pictures in this platform, users need to arrange their DICOM files and specify their intended parameters. DPARSF then will deliver all the preprocessed data as different variety of desirable data for classification. This desirable data consists of slice timing images, normalized images, smooth data, functional connectivity with specific data, ReHo, ALFF/fALFF, degree centrality, and voxel-mirrored homotopic connectivity (VMHC) results [52]. For PET image processing, using a standard CL pipeline is a conventional method [53]. PET images were intensity normalized using the whole cerebellum as a reference region. In simple image preprocessing, the fusion parameters of combination methods have been eliminated.

However, the use of feature selection and normalization part of the procedure remains the same. All of the mentioned algorithms help decrease noise in the picture and use the whole part of the brain, which help model to classify, detect, or recognize ARD. After the acquisition of using complete information, some models will convert pictures into 2D features. With the use of these procedures, the number of features increases significantly. Also, even small shape images like 64*∗*64 or 128*∗*128 have about 4096 or 16384 features. With this amount of information, even power full computational GPU would not conduct the code and render results [54]. So, dimension reduction is a preferable procedure for dealing with image processing tasks. One of the main steps of dimensionality reduction is using correct data and eliminating undesirable data from each picture. Dealing with this task using different norms like l1 and l2 and hybrid classification will help reach a better result. Other studies have used features computed from MRI images to discriminate between different cognitive states related to AD [55]. With the rise in prostate cancer, patient's attention to prostate image segmentation has been conducted. With the use of this data, a semiautomatic method has been designated [56]. This procedure consists of two new algorithms for better feature selection. Experiments on prostate CT images have shown the effect of this method for segmentation and regression tasks [57].

The article "Single and Combined Neuroimaging Techniques for Alzheimer's Disease Detection" was published in 2021. Journal: Comput Intell Neurosci.

Principal Component Analysis (PCA) is another feature selection technique. PCA, in a nutshell, determines the alliance or axis responsible for the most significant amount of variance in the input data set. Respectively, PCA will determine a second axis that must be orthogonal to the first axis responsible for the largest total of remaining data variance. A standard matrix factorization method is called singular value decomposition (SVD) for dealing with this task. This technique will decompose the training data matrix into three different matrices. PCA will be the result of the multiplication of three multiplications. These three matrices will be A, B, and C, where C contains all the principal components used as a principal feature [58]. The whole structure of feature selection and PCA is shown in Figure 8. Effect of proper feature selection and dimension reduction for reaching the better performance of classifier algorithms is necessary. Fewer features will lead to less time consumption in order to train the different models. Using proper features and tuned model state-of-the-art result will be achieved in AD detection and classification.

## 4. Methods

In the last two decades, due to vast improvement of computational power, more conventional GPU and online platforms for the implementation of artificial intelligence (AI) systems have been developed. So, interest in the use of AI, ML, and DL to synthesize the applications for studying mental health has increased rapidly [59]. Different ML algorithms have been used for the prediction and classification of ARD. The main goal of these different algorithms was to separate different patients into AD, MCI, and NC classes [60]. In ML and DL fields, algorithms have been separated into three categories:

- Unsupervised algorithms
- Semisupervised algorithms
- Supervised algorithms

Supervised algorithms refer to algorithms targeting specific targets, and all samples have their target [61]. Most varieties of ML and DL algorithms belong to this category. In this category, gathering samples and labeling them would be tedious. DL can be categorized as a subfield of ML, usually used on big data as input. Different data structures like pictures, time-dependent data, and images can be used for AD classification tasks. It has attracted massive attention in the last few years, especially in image analysis [62]. Several DL architectures such as Convolutional Neural Network (CNN), Deep Neural Network (DNN), Recurrent Neural Network (RNN), and autoencoder (AE) are some examples of these fields which have been used for ARD and classification. Semisupervised learning refers to algorithms that work with a data set that most of its labels are unclear. Most data will be labeled by knowledge about already known labels from data sets [63]. Unsupervised learning refers to algorithms in which labels of the whole data set are not clear. In most cases, most data do not have any labels, making this category very important [64].

The article "Single and Combined Neuroimaging Techniques for Alzheimer's Disease Detection" was published in 2021. Journal: Comput Intell Neurosci.

### 4.1. Semisupervised Methods

#### 4.1.1. K Nearest Neighbor (KNN)

Most used cases of semisupervised learning algorithms rely on Euclidean distances. The famous semisupervised learning algorithms are K Nearest Neighbor (KNN) and its branch [65]. The work structure here is simply finding a cluster of labeled data, computing the average of this cluster, and then computing Euclidean distances of unlabeled data from this mean of labeled data. Finally, labeling data set based on their nearest known average cluster of data will be done. After labeling the data set, supervised algorithms such as CNN or DNN will classify the data set [66]. How semisupervised algorithms will deal with semilabeled data has been shown in Figure 9. Most of the different classification methods will repeat some examples from nature. Semisupervised algorithms will use the procedure of learning in humans. With different years of education, we humans will learn a little labeled information and solve unseen challenges. A variety of different models have been used as a semisupervised algorithm for classification. El-Yacoubi et al. [67] have proposed an approach based on generating each subject cluster and analyzing the correlation of these clusters with NC, AD, and MCI profiles. The main aim of their work was to find the optimal number of clusters and a subset of valuable features that help reach an excellent discriminative algorithm. They used a semisupervised algorithm based on normalized mutual information feature selection, which guides a clustering algorithm to optimize the choice for the number of optimal clusters and the discriminative power of each three-output class. Pohl and Davatzikos [68] used semisupervised algorithms for classification tasks which use both labeled and unlabeled data for training as all semisupervised algorithms do.

The article "Single and Combined Neuroimaging Techniques for Alzheimer's Disease Detection" was published in 2021. Journal: Comput Intell Neurosci.

They used clustering methods to deal with unlabeled data; then, for training the labeled data, they used the linear Laplacian support vector machine (LapSVM) [69]. Gorriz et al. [70] Proposed a novel case-based model selection method at their time, which syndicates hypothesis testing from a separate set of expected results and feature extraction. For the training and validation part, they have used a cross-validation strategy for avoiding overfitting. This proposed model will take advantage of proper feature selection. Using good features, this model tries to improve the network's performance on validation and test sets.

#### 4.1.2. Generative Adversarial Network (GANs)

GANs were first developed and pioneered in 2014 and, from then until now, have gathered much attention on image generation tasks [71]. The use of GANs as semisupervised methods is one of the most capable areas of real-world application of GANs. In a nutshell, semisupervised GAN (SGAN) is a subset of GANs in which discriminator is a multiclass classifier, and its generator is an expanded CNN. Instead of distinguishing between only two classes, it learns to distinguish three or more classes with the production of fake images. Generator in SGAN is not the essential part, unlike other conventional GANs which have aimed to produce new high-quality data from the useless noisy data set [72]. The structure of SGAN has been shown in Figure 10. As shown in Figure 10, the generative part of the network will expand the dimension of noise to create fake images. The SGAN generator's aim is the same as in the original GAN. The generator of ordinal GANs will take a vector of random like Gaussian noise. It will produce fake examples or samples where the goal is very similar to natural images as input data of the training data set. The goal of the generator is the same in SGANs and GANs. The SGAN discriminator, on the other hand, differs obviously from the original GAN procedures. Discriminators of SGANs will get three sorts of inputs: fake examples produced by the generator model, real examples without any labels from the train set, and real examples with labels from the training data. Instead of binary classification, the SGAN discriminator's goal is to distinguish between real and fake examples and then use the labeled data and fake image to classify the input into different classes. In research by Yu et al. [73], the authors used SGAN to predict MCI and AD. They proposed that THS-GAN is designed for semisupervised classification. They have used partially labeled data set input.

The article "Single and Combined Neuroimaging Techniques for Alzheimer's Disease Detection" was published in 2021. Journal: Comput Intell Neurosci.

Then used the distribution of labels to predict the label for both labeled and unlabeled data and the newly generated samples. Their model can profit from the mechanical information of the brain. Also, they introduced high-order pooling, which helps to exploit more essential features by using the second-order statistics of the holistic MRI images. The result of THS-GAN demonstrates that the classification of MCI vs. NC has been done with 89.29% accuracy. AD vs. NC classification has been done with 95.92% accuracy.

### 4.2. Supervised Learning

Supervised methods have higher popularity because of their performance. In this section, supervised methods for AD detection have been reviewed. In real-world data sets, much of the data are not correctly labeled. So, the use of supervised methods will be restricted only to the labeled data set. This review first focused on DL algorithms and then used ML algorithms such as support vector machine (SVM) [74].

#### 4.2.1. DNN

The DNN structure is similar to the traditional multilayer perceptron network structure, and with more perceptron layers, the structure of models will get deeper. This deep model can learn the more sophisticated pattern and relations from input data [75]. The model with a deep layer can determine the best features for classification. DNNs have been used only as supervised methods. We separate the DL method into Conventional Neural Network (CNN), Recurrent Neural Network (RNN), and MLP (Vanilla or Residual Model). 2D CNN is the most used type of CNN for the classification and detection of ARD. The new research focused on using 3D and 4D convolutional layers to extract information from videos [76, 77]. First, we describe CNN because of the common use of this method for AD classification.

#### 4.2.2. Convolutional Neural Network (CNN)

The difference between DNN and CNN methods can be described in the connectivity of neurons in different CNN network layers. The connection in the primarily convolutional layer is not connected to all connections of the second layer. The first layer of convolutional layers extracts simple structure from images like orthogonal and diagonal lines. As the CNN structure goes further and gets deeper complex shapes like face and trapezoid shape can be extracted from images [78]. In each layer of CNN, CNN's top layers are connected to a restricted number of neurons in the next or precious layer located within a specific rectangle shape. This building structure of CNN permits the proposed model to focus on a small sublevel of features in the first hidden layer. Model uses them into more extensive higher-level features in the second hidden layer, and the same structure will be repeated until the last layer. This hierarchical structure is typical in real-world images, like ARD. Complete structural work of CNN consists of the following:

- Specifying the convolutional kernels which are defined by a width and heights
- Specifying the number of input and output channels of each convolutional layer
- Specifying the depth of each convolutional layer must be the same as the number of RGB colors in input data

The structure of CNN consists of a pooling layer that helps whole algorithms work with the smaller size of pictures and have the same performance as full pictures [79]. At the end of the convolutional layer, a flatten layer and stack of multilayer perceptron layers complete the whole structure of CNN. The structure of some CNN is shown in Figure 11.

The article "Single and Combined Neuroimaging Techniques for Alzheimer's Disease Detection" was published in 2021. Journal: Comput Intell Neurosci.

As shown in Figure 11, CNN will increase the number of channels or depth of the input data while decreasing the widths and height of the input picture. The exact location of a feature is less important than its irregular location comparative to other features in the convolutional layer. It is the idea behind the use of a pooling layer in convolutional neural networks. The pooling layer will extract the essential features from the output of convolutional layers. With the pooling layer, the height and width of the input layer will decrease by a factor of the pooling layer's window. The use of the pooling layer will help to reduce overfitting and computational power, which is needed to train the CNN model. After the convolutional layer, a fully connected layer will be used. This model uses MLP as a feedforward network and tries to classify input features [80]. Sarraf and Tofighi [81] used the fundamental type of ordinal CNN called vanilla CNN to exploit different patterns from input data to develop a proper model for AD diagnosis among elderly patients. They proposed a state-of-the-art DL-based procedure to distinguish AD from NC using MRI and fMRI. The use of proposed pipelines was performed on a GPU-based powerful device as the computing platform. They have categorized their input data into three parts of train, test, and validation. Their research use of fMRI data has been used for the first time in the DL model as an application to distinguish between AD, MCI, and NC. Spasov et al. [82] have proposed a DL to classify input data, combining sMRI, demographic, neuropsychological, and APOe4 genotyping pictures as input data for classification tasks. The innovation of their work consists of the DL model, which learns to distinguish between MCI vs. AD and AD vs. NC. All the analyses of this work were performed on a subset of the Alzheimer's Disease Neuroimaging Initiative (ADNI) database. The data set used in their research consists of 785 participants subcategorized as 192 AD, 409 MCI, and 184 NC. Their research found that the most helpful combination of input data included the sMRI images and the demographic, neuropsychological, and APOe4 data. More and more CNN algorithms have been developed for AD classification. For better understanding, the convolutional layer and the effect of each layer at its input are shown in Figure 12. As shown in Figure 12, as the network goes deeper and deeper, more structure of each data set will get extracted and difference between two input pictures will get more precise.

The article "Single and Combined Neuroimaging Techniques for Alzheimer's Disease Detection" was published in 2021. Journal: Comput Intell Neurosci.

#### 4.2.3. RNN with CNN

RNN is a subtype of DNN that remembers earlier time-series data and uses this information with present input for predicting the future. RNN is a structure of time-variant algorithms with repeated information along with its layers.

The min different part of RNN which separates them from other DNN models is the structure of hidden states. This hidden state will help to extract useful information in the sequence of data. The same recurrent layer will be used as a stacked layer after each other. The use of this structure will be helpful in input data as video for the AD classification task. It results in the reduction of the complexity parameters, unlike the other DNN [83]. Two main subcategories of RNN algorithms are Long-Short-Term Memory (LSTM) and Gated Recurrent Unit (GRU). The main purpose of LSTM is to help to use and maintain the error signals through the structure of network models on the long sequence of data.

This maintenance of signal error will be done with short-term memory and long-term memory. The common activation functions used in RNN structure are sigmoid and tanh, which can help backpropagate error signal through different layers. In LSTM, different gates will be used for the preservation of information and ignoring redundant information. These gates consist of learning gates, forget gates, use gates, and remember gates. LSTM model is similar to a computer's memory. This cell's structure can be used independently to decide which information to store and which information to forget [84]. The structure of the RNN and LSTM network is shown in Figure 13. As shown in Figure 13, the LSTM structure is more complex, but the flow of loss throws each layer for a better optimization process. Karlekar et al. [85] had used language changes as a sign of a patient's cognitive functionality for early diagnosis of AD. In their work, they have used Natural Language Processing (NLP) for AD classification tasks. In the proposed work, they have used CNN, LSTM\RNN to distinguish between language samples from AD and other stages of AD. They have reached 91.1% accuracy with this newly conducted procedure.

The article "Single and Combined Neuroimaging Techniques for Alzheimer's Disease Detection" was published in 2021. Journal: Comput Intell Neurosci.

#### 4.2.4. Machine Learning Algorithm

The use of supervised ML algorithms for classification is not more different than a semisupervised algorithm for classification. The difference between these two algorithms appears in part of the labeling data set. For a supervised classifier, all data labels are specified, but in semisupervised one, all data labels are not clear. A method that has been used for a handful of researches is SVM. In research by Kloppel et al. [86], they used SVM with the linear kernel to classify MRI scans from proven AD patients and MCI in elderly cases with two different scanning equipment and neuroimaging techniques. Finally, they used these methods to differentiate between patients suffering from AD and patients with frontotemporal lobar degeneration. The result of the classification models consists of 89% accuracy. In another research by Montagne et al. [87], they proposed a model based on a noninvasive neuroimaging technique for early diagnosis of ARD. They have used SVM to classify Alzheimer's disease versus NC group of patients. They have reached better classification rates by focusing on parietal and temporal lobes of brains with SVM. Other ML methods used for AD classification comprise using second-order derivation or Hessian of loss function for updating weight. Extreme Learning Machine (ELM) is another popular algorithm for classification too.

ELM is a learning algorithm conducted without using multiple different stacked layers and tuning this vast majority of hidden layer and input so that the computation time will decrease [87]. In ELM, unlike other DNN algorithms and SVM, the hidden layer parameters consist of weights and biases. One hidden layer does not need to be tuned after importing the data set and can be generated randomly before the training samples are acquired. This modification will help the network for faster learning processes at the cost of higher loss [88]. In an article by Lama et al. [89], they proposed an AD diagnosis approach using sMRI images to discriminate AD, mild MCI, and NC. They have used SVM and a regularized ELM for prediction. Lama et al. experimented on the ADNI data sets. They showed that regularized ELM with the feature selection techniques could significantly improve the classification accuracy of AD from MCI and NC subjects.

## 5. Comparison Based on the Different Types of Data

### 5.1. fMRI, sMRI, and rs-fMRI

In this section use of different algorithms based on fMRI and sMRI pictures has been surveyed. In research by Duc et al. [7], different variants of MRI like sMRI and rs-MRI scans of 331 subject patients for Mini Mental State Examination prediction have been used. In their work, 3-dimensional CNN, a method, has been developed for the mentioned classification task. Task linear regression, support vector regression, bagging-based ensemble regression, and tree regression were used. They have reached a test accuracy of 85.27% for the classification of AD versus NC. Also, it was mentioned that the SVM method with desired features has reached the lowest root mean square error of 3.27 and the highest R2 value of 0.63. As seen from this work structure, a perfect relation between input data and regression task had not been reported.

The article "Single and Combined Neuroimaging Techniques for Alzheimer's Disease Detection" was published in 2021. Journal: Comput Intell Neurosci.

In another research, Ramzan et al. [90] have studied the effect of rs-fMRI for multiclass classification of AD and different stages of AD-related disease. They have used one of the famous structures of CNN, which is ResNet-18 [91]. The mentioned structure consists of skip connection for better use of error signal in backpropagation technique for optimization. Skip connection will help the model to get deeper with the vanishing of gradient signals. They have conducted model training from scratch with single-channel input. On the other hand, they also have performed transfer learning with and without an extended network architecture. Transfer learning helped them reach a state-of-the-art result with an average accuracy of 97.92% and 97.88% for all the AD stages prediction. Altinkaya et al. [92] have used superresolution on the low quality of input MRI picture and then used CNN for AD prediction. With superresolution, image processing time has been shortened, and images with high-quality features have been obtained. The result of their study concluded that the performance of proposed methods increased day by day. The resulting accuracy with CNN for AD detection using 302 MRI and fMRI instances was 99.9%.

Korolev et al. [93] have used 3DCNN and achieved better performance without including preprocessing steps like feature extraction in their proposed architecture. These proposed methods consist of CNN and the residual NN. In terms of performance metric Area under Receiver Operating Characteristic (AROC), receiver operating characteristics (ROC) curves, and accuracy have been evaluated. They have proposed a branch of CNN which is called Vox CNN and ordinal ResNet. AD vs. NC achieved the best result with AUC 0.88 and acc 0.79 using VoxCNN and AUC 0.87 with acc 0.80 using ResNet.

The article "Single and Combined Neuroimaging Techniques for Alzheimer's Disease Detection" was published in 2021. Journal: Comput Intell Neurosci.

Li et al. [94] have used hippocampal MRI as input data. They surveyed 2146 subjects for prediction of MCI in each subject and how this stage will progress and lead to dementia in a time-to-event analysis setup. This study focused on the hippocampus region of the brain. They have reached 0.813 AUROC. For better results use of whole-brain MRI data can help different DL models to reach better classification tasks.

Yang et al. [95] have used SGANs with clustering as the novel semisupervised deep-clustering method. They have surveyed 8,146 scans which included NC, those with MCI, and dementia cognitively. One-fourth of their input data consists of sMRI data. Their proposed method has separated patients into four types of peoples: NC, MCI, relatively more significant memory impairment, and advanced dementia. Results of their work confirmed that the Smile-GAN model was able to cluster participants with 99.9% accuracy even with very severe confusing patterns as inputs. Zeng et al. [88] have proposed a total baseline for the diagnosis of AD. Their proposed model consists of MRI image preprocessing, feature extraction, PCA, and SVM algorithm developments at the end. For optimization, a particle swarm optimization algorithm was proposed to optimize the SVM parameters instead of traditional optimization methods. With their proposed model, they successfully conducted a classification of AD and MCI using MRI scans from the ADNI data set. The proposed algorithm in their research has a state-of-the-art performance compared to other presented methods [87]. Dua et al. [96] used MRI scans from different online repositories to create a diverse data set. They have deployed CNN, RNN, and LSTM individually and as ensemble methods together. The results of the proposed work show that, with the combination of CNN with RNN and CNN with LSTM, an accuracy of 89.75% has been achieved. Meanwhile, they have also used ensemble method with the bagging strategy of the first models. They achieved an accuracy of 92.22%. According to the structure of video and 4D, CNN's use of RNN with this specific data structure has shown promising results [97]. It has been shown that use of 3DCNN and stacked bidirectional LSTM could help the researcher to reach state-of-the-art performance based on accuracy and loss [97]. In research by Kruthika and Maheshappa [76], a DNN has used capsule networks, a branch of CNN. This method will use the benefit of not using any max-pooling layers. The structure of the capsule net has been developed to use spatial information in the pictures. They have proposed a 3DCNN, which works with video structure too. Their work proposed a method based on CNN and capsule networks for AD prediction using MRI data as input. In the end, they have used the proposed model for creating an application for the AD detection task. They found that both the 3D capsule network method and CNN with pretrained 3D autoencoder improved the predictive performance compared to other structures of CNN trained from scratch. In another research, multiclass classification between AD, MCI, and NC has seen a state-of-the-art CNN called MCADNNet [98]. Using the mentioned method, the researcher reached 92.6% accuracy with distinguishable accuracy of 97% for MCI classification versus AD subjects. Furthermore, even after applying the decision-making algorithm, accuracy rates of 99.77% and 97.5% were achieved for MRI and fMRI pipelines to classify AD versus NC. Amini et al. [99] used CNN and ML models for finding the severity of AD. They have used fMRI pictures as input data set. Also, they have used a sophisticated procedure for converting raw fMRI input data into a valuable data set for training CNN and ML models. The performance of the proposed CNN model for different stages of AD classification was 98.1%, 92.4%, 97.0%, and 100% precision for the low, mild, moderate, and severe status of Alzheimer's patients. The absolute accuracy for their work was reported at 96.7%. They have used only vanilla CNN with one convolutional layer and three fully connected layers. Mentioned structure without any pooling layer is a variant of CNN, which helps to extract features from low dimension feature maps [100].

The article "Single and Combined Neuroimaging Techniques for Alzheimer's Disease Detection" was published in 2021. Journal: Comput Intell Neurosci.

### 5.2. PET

The use of PET as a biomarker for AD-related detection is a relatively new procedure. Ozsahin et al. [101] have proposed amyloid-beta plaques combination as a marker. They have implied that mentioned marker should be taken for granted as a “start” of the degenerative process in the brain of most cases. This symptom can be seen earlier than other clinical symptoms, which will appear later in AD subjects. They have used DNN with 18F-florbetapir PET data for automatic classification of four patient groups into four different classes of people, which consist of the following:

- AD
- Late MCI
- Early MCI
- Significant memory concern
- NC

With this specification, even early stages of AD disease can be detected. Their work on 30% of data as test cases based on sensitivity, specificity, and accuracy was measured as 92.4%, 84.3%, and 87.9%, respectively. Other parts of the second experiment, which consist of the classification of NC versus late MCI images, resulted in sensitivity, specificity, and accuracy of 62.9%, 70.0%, and 66.4%. Other experiments in the classification of NC versus early MCI images have shown the sensitivity of 60.0%, specificity of 60.0%, and accuracy of 60.0%. Finally, NC has significant memory concern as other classes have been used for classification, and the result of their work showed sensitivity, specificity, and accuracy values of 60.0%, 45.7%, and 52.9%.

The article "Single and Combined Neuroimaging Techniques for Alzheimer's Disease Detection" was published in 2021. Journal: Comput Intell Neurosci.

The use of ML for improving AD detection in the analysis of digital biomarkers within PET imaging has emerged recently. Islam et al. [102] have proposed a 3DCNN for AD diagnosis using only PET scans. They have reached the classification accuracy of 88.76% for NC versus AD categories. Their experiment also developed a regular CNN model using axial, coronal, and sagittal segments from each subject's brain from PET data; in the end, they have achieved 71.45% accuracy for NC versus AD classification.

In another research by Vasan et al. [103], F-FDG-PET brain images from the ADNI repository have been used to train the models for testing the result of the training model; they have used an independent test set from individual patients. They have used a branch of CNN which is called InceptionV3 [104]. Using this model, they reached AUC to predict AD, MCI, and NC, of 92%, 0.63%, and 0.73%, respectively. The AUROC for this classification task was 0.98, 0.52, and 0.84 to predict AD, MCI, and NC, respectively. The reported sensitivity consists of 100%, 43%, and 35% for AD, MCI, and NC prediction, respectively. As it is shown, the best result has been achieved for AD classification.

Lu et al. [105] used Fluoro-deoxy-glucose positron emission tomography (FDG-PET) to detect the brain's metabolic activity in the different subjects as data set. They proposed a novel DL method at the time for analyzing the FDG-PET. They used this information to classify MCI subjects with symptomatic AD and distinguish them from other subjects with MCI stages. The result of their work shows 82.51% accuracy of classification just using measures from a single modality. Because of the similarity between these two stages, their work can distinguish between two similar stages rather than AD versus NC.

Adeli et al. [106] proposed a semisupervised algorithm for first dealing with little labeled data and the vast majority of unable data. The discriminative classification method based on the least-squares formulation of linear discriminant analysis has been used in work. The use of a linear discriminant model has helped them to deal with noisy and unwanted data. They have surveyed Parkinson's and AD diseases as neurodegenerative diseases. They have used their framework to create an application for neurodegenerative disease diagnosis. They have reached 92.1% accuracy for AD versus NC classifications. In another work by Gamberger et al. [105], they have analyzed 5-year longitudinal outcomes and biomarker data from 562 subjects with MCI from ADNI. The mentioned algorithm identified homogenous clusters of MCI subjects with evidently diverse predictive cognitive courses. In the end, they have reported high sensitivity and specificity for the classification of AD versus NC.

The article "Single and Combined Neuroimaging Techniques for Alzheimer's Disease Detection" was published in 2021. Journal: Comput Intell Neurosci.

In another research by Liu et al. [107], they used FDG-PET data as input for training. They have used DL models with the combination of GRU and convolutional layers. Their proposed model has abled them to use intrasegment and intersegment to classify different stages of AD disease. They have used the different frames of video and then developed a CNN model on these images. In the structure of the proposed model, the convolutions layer has been used only to capture the valuable features from input image data. After reaching good data, they used GRU and RNN to learn and integrate the intersegment features for classification tasks. They reached 95.3% for AD versus NC classification and 83.9% for MCI versus NC classification based on AUC metrics. Their proposed method reached 91.2% accuracy, 91.4%sensitivity, and 91.0 specificity for AD versus NC condition, respectively.

### 5.3. Combination of Data

Combining PET and different branches of MRI data with the aim of reaching a diverse data set with complementary effects has gained attention. Gupta et al. [35] have used a combination of four different biomarkers: FDG-PET, sMRI, the level of protein in cerebrospinal fluid (CSF) data, and apolipoprotein (APOE) genotype. They have used data set from ADNI as their baseline data set. In total, they have surveyed 158 patients whose all of the mentioned input data are available for each of these subjects. In their study, patients were divided into 38 subjects of AD, 82 subjects of MCI groups, and the remaining 38 subjects in the NC group. With these categories of data set, their data set was imbalanced. They used a kernel-based multiclass SVM classifier with a grid-search method and truncated PCA to determine the best feature to use for training. They have reached AUROC 98.33%, 93.59%, 96.83%, 94.64%, 96.43%, and 95.24% for AD versus NC, MCIs versus MCIc, AD versus MCIs, AD versus MCIc, NC versus MCIc, and NC versus MCIs classification. The accuracy, sensitivity, and F1-score of AD and NC classification were 98.42%, 100%, and 98.42%. The result of their work has shown some state-of-the-art results for AD classifications. The result of their work has shown a significant rise in accuracy in different stages from previous works.

Youssofzadeh et al. [34] used MRI and PET in combination due to their complementary nature as the input data set. They have used a multimodal imaging ML to enhance AD classification performance metrics. They have used 58 AD subjects, 108 MCI subjects, and 120 NC subjects from the Australian imaging, biomarkers, and lifestyle data set. For classification of AD versus NC, MCI versus NC, and AD versus NC, they reached 95.7%, 95.8%, and 95.1% accuracy, respectively. Also, they have found multikernel learning regression analysis for excellent predictions of diagnosis of AD in subjected samples with a relation factor of 0.86. In addition, they have reached significant correlations between developed methods and delayed memory recall scores with a relation factor of 0.62.

The article "Single and Combined Neuroimaging Techniques for Alzheimer's Disease Detection" was published in 2021. Journal: Comput Intell Neurosci.

In another research, Li et al. [108] used whole-brain images as input and designed a disease-image-specific neural network for the classification task of AD subjects. They have used MRI and PET scans as input data for classification tasks. Also, they have used feature-consistent GANs to produce some images for better results of classification. Using this branch of GAN, they have encouraged the proposed model to use these produced images and authentic images as a consistent data set for final prediction. Their work conducted a state-of-the-art performance in both AD identification and MCI conversion prediction tasks at times. They have reached 34.18% in terms of the PR-AUC score.

In another study, Dukart et al. [109] used MRI and fluorodeoxyglucose FDG-PET to improve the detection accuracy of differentiation subjects with AD complication and frontotemporal lobar neuron connection failure. They have used an SVM classifier for this task. SVM classification has used combined information from different ROI of each subject from FDG-PET and MRI based on comprehensive quantitative meta-analyses. For the ADNI data set, accuracy rates of 88% have been achieved. In another work by Triebkorn et al. [110], they have used an amyloid-beta marker from each PET data from each patient. Also, they have used MRI, specifically amyloid-beta binding tracer PET, and tau protein (Tau) binding PET from 33 participants of ADNI3. Their work aims to classify AD MCI and NC using SVM and Random Forest classifiers together. They have reached 90.5% accuracy for NC versus AD and MCI classification. For AD versus NC and MCI classification, they have reached 78.3% accuracy. The sensitivity of this classifier method for NC versus AD and MCI classification was 90.5%. They also have reached AD versus HC and MCI classification of 78.3%.

In research by Kim and Lee [111], they proposed an autoencoder and sparse ELM to classify AD versus NC and MCI. They have used MRI, PET, and CSF pictures from 93 individual subjects. They have extracted volume and means ROIs as input features. At last, they have used a stacked sparse ELM autoencoder for the classification task. The use of an autoencoder for changing the input space into smaller later space has been done. For evaluating the proposed model, they have used 10-fold cross-validation. The classification result has shown more than 96% and 86.44% accuracy for classifying AD versus NC and MCI versus NC subjects.

The article "Single and Combined Neuroimaging Techniques for Alzheimer's Disease Detection" was published in 2021. Journal: Comput Intell Neurosci.

### 5.4. Comparison between Different Modalities

In this section, we compared different neuroimaging modalities according to their performance. Comparison has been made based on different metrics such as accuracy, precision, recall, F1-score, and area under the receiver AROC. Accuracy is given in the following:

(1) $$\begin{array}{c} \text{sensitivity}=\left[\frac{\text{TP}}{\text{TP}+\text{FN}}\right]\times 100,\\ \text{specificity}=\left[\frac{\text{TN}}{\text{TN}+\text{FP}}\right]\times 100,\\ \text{positive predictive value}\left(\text{PPV}\right)=\left[\frac{\text{TP}}{\text{TP}+\text{FP}}\right]\times 100,\\ \text{negative predictive value}\left(\text{NPV}\right)=\left[\frac{\text{TN}}{\text{TN}+\text{FN}}\right]\times 100,\\ \text{accuracy}\left(\text{ACC}\right)=\left[\frac{\text{TP}+\text{TN}}{\text{TP}+\text{TN}+\text{FP}+\text{FN}}\right]\times 100. \end{array}$$

Based on mentioned metrics, an evaluation of binary and multiclass classification can be done. As shown in Table 1, different methods used MRI as input data. Most of them have reached a good accuracy too. Using PET as data set for the sake of AD detection only based on accuracy is lower than MRI as input. Combined modalities have shown better performance based on accuracy than single data. The best algorithms for prediction consist of a different branch of CNN.

## 6. Results

Alzheimer's disease is the main cause of memory loss and dementia in people older than 65. AD consists of a gradually progressive neurodegenerative disease process consisting of gradual synaptic integrity and loss of cognitive functions. For detecting AD, a marker as a sign of progressive neurodegenerative is needed. This marker has a more critical role for AD detection than other diseases because beta-amyloid can form a complex structure with some metal ions. For assessing this marker, some neuroimaging techniques like fMRI and sMRI, PET, PET (FDG), and combination of these data have been used (see Table 1).

AI and its branches have helped with AD detection in patients with various methods. Some of these algorithms consist of ANN, CNN, and GANs as supervised and semisupervised algorithms. Other famous ML algorithms such as KNN, SVM, and RF have been used too. This review article discussed different neuroimaging techniques and has shown some effects of some of the DL methods on this input data for AD detection. In the end, we have to summarize these different techniques and compare them based on accuracy, sensitivity, and AUROC. The results showed that combined neuroimaging techniques are a newly open field, and DL methods for detecting AD on average are of high accuracy. For people older than 65, if we want a model to be sensitive and its prediction considers low false-negative outcomes, MRI and CNN base methods have shown better results. In full use of the combination, methods have much more unspecific areas for research. As shown in Table 1 more than half of the reviewed article was published in 2020 and 2021. This year's focus on GANs and using VGG and resent structure with combination data from different repositories have gained more attention. Some articles have reached 99% accuracy with old popular CNN for AD versus NC classification task only. With proceeding years, using different methods for reaching a good accuracy has paid off, and most of the articles have reached a state-of-the-art accuracy. The result of accuracy versus years is shown in Figure 14. Time-series signals related to specific parts of the brain as input data and use of CNN or ML models for AD classification are another center of attention for researchers [100, 127]. As discussed, we focused on AD versus NC classification improvements as the main priority. The reputation of authors or the number of citations for each research has not been considered in this article.

The article "Single and Combined Neuroimaging Techniques for Alzheimer's Disease Detection" was published in 2021. Journal: Comput Intell Neurosci.

## 7. Conclusion and Discussion

Different ML techniques for AD classification and detection have been reviewed in this article. For gathering different images, data time consumption and the financial issue should be considered. Also, the use of combined data has shown promising performance. So, this is a trade-off that should solve this. Most of the research has worked on the ADNI data set due to its convenient access and variety of stages of the data set. AD versus NC and MCI classification has been surveyed in most of the researches. The use of different data set will add more controversy and variety to the data set. This variety is an essential part of each data set. So, for better and more comprehensive results use of a different variety of data must be considered. Also, for better early AD detection, different AD stages as a data set should be considered.

## Figures and Tables

**Figure 1:** Example of magnetic resonance imaging (MRI).

**Figure 2:** Example of functional magnetic resonance imaging (fMRI) in different stages. (a) Slice number: 0. (b) Slice number: 10. (c) Slice number: 20. (d) Slice number: 30.

The article "Single and Combined Neuroimaging Techniques for Alzheimer's Disease Detection" was published in 2021. Journal: Comput Intell Neurosci.

**Figure 3:** Example of fMRI in different stages.

**Figure 4:** Example of rs-fMRI in different stages. (a) Slice number: 0. (b) Slice number: 10. (c) Slice number: 20. (d) Slice number: 30.

**Figure 5:** Example of PET in different stages. (a) Slice number: 0. (b) Slice number: 20. (c) Slice number: 40. (d) Slice number: 60. (e) Slice number: 80. (f) Slice number: 100. (g) Slice number: 120. (h) Slice number: 140. (i) Slice number: 160. (j) Slice number: 180.

**Figure 6:** Combination of PET with rs-fMRI pictures.

**Figure 7:** Combination of PET with rs-fMRI pictures in the processing of data preprocessing.

**Figure 8:** Diagram of feature selection and PCA.

**Figure 9:** Semisupervised learning method for binary AD classification.

**Figure 10:** Semisupervised GAN learning method for binary AD classification.

**Figure 11:** Structure of CNN.

**Figure 12:** Result of convolutional layer on input image for (a) first convolutional layer, (b) second convolutional layer, and (c) last convolutional layer.

**Figure 13:** Structure of (a) RNN versus (b) LSTM.

**Figure 14:** Different accuracy based on different years.

**Table 1:** Summary of methods and neuroimaging techniques for binary classification of AD versus NC results.

Num.	Reference	Year	Method data	Neuroimaging	Accuracy	Sensitivity	AUROC
1	Duc et al. [7]	2020	3DCNN	rs-fMRI	85.27%	—	—
2	Ramzan et al. [90]	2020	CNN (ResNet-18)	fMRI	97.88%	—	—
3	Altinkaya et al. [92]	2020	CNN	fMRI	99.9 (on 303 samples)	—	—
4	Korolev et al. [93]	2017	CNN (ResNet)	MRI	80%	—	0.87
5	Li et al. [101]	2019	CNN	MRI	—	—	0.82
6	Yang et al. [95]	2021	GANs	MRI	99%	—	—
7	Dua et al. [96]	2020	CNN-LSTM (RNN)	MRI	92.22%	91.92%	
8	Zeng et al. [88]	2018	CNN (PSO)	MRI	76.85%	—	—
9	Kruthika and Maheshappa [76]	2019	3DCNN (capsule net)	sMRI	92.98%	—	0.98
10	Sarraf et al. [112]	2019	CNN (MCADNNet)	fMRI + MRI	99%	95%	—
11	Ozsahin et al. [102]	2019	ANN	PET	87.9%	92.4%	—
12	Islam and Zhang [113]	2019	3DCNN	PET (FDG)	88.76%	—	—
13	Vasan et al. [103]	2020	CNN (Inceptionv3)	PET	92%	100%	0.98
14	Lu et al. [105]	2017	ANN	PET (FDG)	82.51%	—	—
15	Adeli et al. [106]	2018	RF	PET	92%	—	0.94
16	Liu et al. [110]	2021	CNN-RNN (GRU)	PET	91.2%	92.4%	0.94
17	Gupta et al. [34]	2017	SVM	PET + MRI	92%	98.42%	0.98
18	Youssofzadeh et al. [109]	2013	MKML	PET + MRI	95.7%	—	—
19	Li et al. [108]	2018	GANs	PET (FDG) + MRI	—	—	0.32
20	Dukart et al. [107]	2018	SVM	PET (FDG) + MRI	78.3%	90.5%	—
21	Kim and Lee [111]	2018	ANN (AE)	PET (FDG) + MRI	96%	—	—
22	Billones et al. [114]	2016	CNN (DemNET)	MRI	98.33%	98.99%	—
23	Talo et al. [115]	2019	CNN (DeepResNet-50)	MRI	95.23%	97.16%	—
24	Yu et al. [73]	2020	THS-GAN	MRI	95.92%	—	—
25	Moradi et al. [116]	2015	Semisupervised model	MRI	87%	82%	
26	Kloppel et al. [86]	2004	SVM	MRI	88%	—	—
27	Montagne et al. [87]	2013	SVM	PET	82%	81%	—
28	Lama et al. [89]	2017	ELM	Smri	83.38%	93.01%	0.85
29	Lin et al. [117]	2021	GANs + 3D VGG	PET (FDG) + MRI	74.1%	75.00%	0.92
30	Zhou et al. [118]	2021	GANs + DNN	MRI	88.73%	63.09%	0.932
31	Baydargil et al. [119]	2021	GANs	PET	96.03%	—	0.7521
32	Venugopalan et al. [120]	2021	DNN + RF	PET + MRI	89%	96%	—
33	Zhang et al. [121]	2021	3DCNN	MRI	97.35%	97.10%	0.9970
34	Mehmood et al. [122]	2021	CNN	MRI	98.73%	—	—
35	Raju et al. [123]	2021	CNN (VGG16 based model)	MRI	99.2%	98.5%	—
36	Subramoniam [124]	2021	CNN (ResNet 101)	MRI	99.71%	0.99	1
37	Lella et al. [125]	2021	ELM	MRI	89.25%	0.78	—
38	Acharya et al. [126]	2019	KNN	MRI	94.54%	0.96	—
39	Amini et al. [99]	2021	SVM + PCA	fMRI	85.8%	0.95	0.92
40	Amini et al. [99]	2021	KNN + PCA	fMRI	77.5%	0.98	0.93
41	Amini et al. [99]	2021	CNN	fMRI	96.7%	0.98	1

The article "Single and Combined Neuroimaging Techniques for Alzheimer's Disease Detection" was published in 2021. Journal: Comput Intell Neurosci.

## Data Availability

Data used in this paper's preparation were obtained from the ADNI database (http://adni.loni.usc.edu/).
